The article "A Review of Detection of Antibiotic Residues in Food by Surface-Enhanced Raman Spectroscopy" was retracted in 2024. Reasons: signs of a paper mill; suspected computer-generated content; unreliable results or conclusions; concerns about the data.

# A Review of Detection of Antibiotic Residues in Food by Surface-Enhanced Raman Spectroscopy

**DOI:** 10.1155/2021/8180154

**Published:** 2021-11-05

**Authors:** Jun-Fa Liang, Cheng Peng, Peiyu Li, Qiu-Xiong Ye, Yu Wang, Yun-Ting Yi, Zi-Sheng Yao, Gui-Yun Chen, Bin-Bin Zhang, Jia-Jian Lin, Qizhi Luo, Xuncai Chen

**Affiliations:** ^1^Guangzhou Institute of Food Inspection, Guangzhou, China; ^2^Department of Forensic Toxicology, School of Forensic Medicine, Southern Medical University, Guangzhou 510515, China; ^3^Guangzhou Key Laboratory of Forensic Multi-Omics for Precision Identification, School of Forensic Medicine, Southern Medical University, Guangzhou 510515, China

## Abstract

Antibiotics, as veterinary drugs, have made extremely important contributions to disease prevention and treatment in the animal breeding industry. However, the accumulation of antibiotics in animal food due to their overuse during animal feeding is a frequent occurrence, which in turn would cause serious harm to public health when they are consumed by humans. Antibiotic residues in food have become one of the central issues in global food safety. As a safety measure, rapid and effective analytical approaches for detecting these residues must be implemented to prevent contaminated products from reaching the consumers. Traditional analytical methods, such as liquid chromatography, liquid chromatography mass spectrometry, and capillary electrophoresis, involve time-consuming sample preparation and complicated operation and require expensive instrumentation. By comparison, surface-enhanced Raman spectroscopy (SERS) has excellent sensitivity and remarkably enhanced target recognition. Thus, SERS has become a promising alternative analytical method for detecting antibiotic residues, as it can provide an ultrasensitive fingerprint spectrum for the rapid and noninvasive detection of trace analytes. In this study, we comprehensively review the recent progress and advances that have been achieved in the use of SERS in antibiotic residue detection. We introduce and discuss the basic principles of SERS. We then present the prospects and challenges in the use of SERS in the detection of antibiotics in food. Finally, we summarize and discuss the current problems and future trends in the detection of antibiotics in food.

## 1. Introduction

Antibiotics are a class of secondary metabolites or synthetic analogs that not only can interfere with cell development at low concentrations but also kill or inhibit the growth of microorganisms (bacteria, archaea, viruses, protozoa, microalgae, and fungi) [1]. Since Sir Fleming first discovered that penicillin has antibiotic properties in 1928, various antibiotics have been developed and used to prevent and treat human diseases. They have also been widely used in the prevention and treatment of diseases in the animal breeding industry to increase productivity. However, after decades of ubiquitous use of antibiotics, the negative impact of antibiotics on human health and the ecological environment has gradually attracted people's attention and has become a global public concern.

As shown in Figure 1, antibiotics are popularly used in various industries, such as aquaculture, livestock production, poultry production, and agriculture, to increase economic productivity. Antibiotic residues are frequently detected in multiple food products, such as meat, fish, milk, eggs, and fruit. These residues bioaccumulate in the human body through the food chain and then cause damage to human organs, resulting in anemia and cardiovascular diseases [2]. Excessive amounts of antibiotics can also cause bacterial resistance, which would lead to a decrease in the therapeutic efficacy of drugs and cause great harm to human health. In the absence of effective treatment measures, the global death toll is expected to increase to 10 million per year by 2050 because of antibiotic resistance [3]. In view of the toxicity of antibiotics, the Codex Alimentarius Commission has revised maximum residue limits and recommended risk management for residues of veterinary drugs in foods in 2018. Various antibiotics with high toxicity, such as quinolones, are forbidden for use in food animal production.

Most of the previous studies on antibiotics conducted qualitative and quantitative analyses of antibiotics. Antibiotics are detected using traditional detection technologies, such as chromatography and its combined technology [4], capillary electrophoresis [5], immunochromatography [6], and microbiology techniques [7]. As shown in Table 1, these methods can achieve satisfactory sensitivity and accuracy. However, they have attendant disadvantages: they require expensive analytical instruments, sample preparation is time consuming, and operators must be intensively trained. Capillary electrophoresis has low sensitivity and poor reproducibility, as it largely depends on the sample components it can detect. Immunochromatography, a qualitative or semiquantitative detection method, results in a high false-positive rate. Antibiotic detection via various techniques in microbiology are also time consuming. The test results are analyzed by highly trained professionals with their naked eye, which would inevitably lead to inaccurate interpretation of the results.

Surface-enhanced Raman spectroscopy (SERS) is a surface-sensitive technique that enhances Raman scattering by molecules adsorbed on rough metal surfaces. It has been recently developed and applied in antibiotic detection. SERS requires low sample consumption, has a fast response, involves nondestructive and noninvasive analysis, and has good specificity. Moreover, the ability of SERS to analyze the composition of a mixture at the nano scale makes it beneficial for environmental analysis, pharmaceuticals, material sciences [14], drug and explosive detection, and food quality analysis [15].

With the deepening of research involving the use of SERS over the past few decades, various substrates for Raman signal enhancement and different quantitative detection strategies have been developed and used in food safety evaluation [16]. However, most of the previous works focused on pesticide residues [17] and environmental testing [18], and studies on antibiotic detection in food using SERS are few. Therefore, latest research on the application of SERS in antibiotic detection in food must be reviewed to provide a reference for researchers. In this review, we briefly discuss the basic principles of SERS. We examine current advances in the development of active SERS substrates. We summarize the quantitative methods for detecting antibiotics in food and emphasize the roles of sample pretreatment, chemometrics, and functional integration. We assess the current problems encountered in antibiotic detection and explore future research trends in this endeavor. A pathway chain summarizing the use of antibiotic drugs from the breeding industry/agriculture to food products and the implementation of SERS for testing food to prevent humans from consuming food contaminated with antibiotics is depicted in Figure 1.

## 2. Theoretical Basis of SERS

Raman scattering is the inelastic scattering that occurs when photons interact with molecules. According to the classical Raman scattering theory, the efficiency of Raman scattering depends on differential Raman cross section. In general, the Raman scattering cross section of a molecule ranges from 10^−31^ cm^−2^ sr^−1^ to 10^−29^ cm^−2^ sr^−1^ (where sr is sphericity), which is considerably lower than the fluorescence scattering cross section (10^−16^ cm^−2^ sr^−1^) [19]. Therefore, the Raman scattering effect is a very weak process, and the scattering signal that can be detected is only about 10^−10^ of the intensity of incident signal. As a detection technique, the sensitivity of Raman spectroscopy is obviously very low. In addition, owing to the interference of the fluorescence background of samples, Raman spectroscopy cannot readily analyze trace targets, thereby restricting its development in the fields of trace detection and surface science [20].

In 1974, Fleischmann et al. [21] first discovered that the Raman signal of pyridine increased by 10^6^ times over a silver electrode with a rough surface. Thus, discovery laid the foundation for the development of SERS. On the basis of the research by Fleischmann et al., Jeanmaire and Van Duyne [22] and Albrecht and Creighton [23] conducted in-depth explorations of the Raman signal of pyridine. They confirmed that pyridine adsorbed on a silver electrode can substantially increase the intensity of its Raman signal. They extended their research to other nitrogen heterocycles and amines. The discovery of the SERS effect has provided an effective solution to the inherent problems of Raman spectroscopy, namely, low sensitivity, difficult signal acquisition, and strong fluorescent background in surface science and trace analysis. Furthermore, this discovery has opened the door to the application of Raman spectroscopy in various fields.

Numerous studies have been conducted on the surface enhancement mechanism of Raman spectroscopy. However, research on the theoretical basis of SERS relatively lags behind that on its application. The primary bottleneck is the fact that the system of the SERS effect is quite complicated, and many factors influence the intensity of SERS signals, such as the surface morphology of the system, its electronic structure, interactions between photons and rough surfaces, and interactions between photons and molecules [24].

On the basis of specific experimental conditions, scientists have proposed different SERS mechanisms from various perspectives. In general, two basic mechanisms are recognized, namely, electromagnetic field enhancement and chemical enhancement [26]. The illustration of SERS mechanism is shown in Figure 2 [25]. Electromagnetic enhancement (EM) is the dominant mechanism of the surface enhancement Raman effect. In EM, the surface of a metal nanostructure is excited to generate localized plasmon resonance when irradiated with incident light, the specific frequency of which resonates with the incident light. The incident field and the Raman scattering field are then amplified to form a highly concentrated “hot spot” [27]. Chemical enhancement (CM), also known as the “first layer” effect, is the chemical interaction between metal nanoparticles and molecules adsorbed on the surface of a metal. Electrons transfer from the Fermi level of the metal to the lowest unoccupied molecular orbital of the molecule, forming an electron transfer intermediate with a Raman cross section higher than that of a free molecule. Under the photoelectric field effect, the frequency of incident photon resonates with the electron transfer transition of the intermediate, thereby increasing the Raman scattering intensity of the molecule [28]. The mechanisms of CM could be explained by the following factors [29]: (1) nonresonant enhancement due to the chemical bonding between adsorbed molecules and metal substrate, (2) resonance enhancement due to the surface complexes formed by adsorbed molecules and surface-adsorbed atoms, and (3) resonance-like enhancement of light-induced charge transfer in a molecule-metal system by excitation light. In general, in a Raman system, these CM mechanisms work synergistically. The enhancement factor of the chemical bond effect can contribute up to 10^3^, whereas the enhancement factor of the charge transfer effect generated when the electron is excited between the adsorbed molecule and the metal can be up to 10^4^ [30]. CM and EM coexist in most SERS systems.

## 3. Detection of Trace Amounts of Antibiotics in Food via SERS

### 3.1. Active SERS Substrate

An active SERS substrate is a key component of highly sensitive SERS detection [31]. Along with the development of nanotechnology, various active SERS substrates with a high activity have been developed (Table 2). According to differences in their chemical compositions, they can be roughly divided into noble metals, hybrid materials of noble metals and semiconductors, and hybrid materials of noble metals and metal-organic frameworks (MOFs) [56]. In the following section, latest research on different SERS substrates is discussed.

#### 3.1.1. Noble Metals as Active SERS Substrates

The SERS performance of noble metal nanomaterials largely depends on their size, morphology, composition, and structure. Noble metal nanomaterials with different morphologies, such as gold nanostars [57], silver nanodendrites [58], flower-like gold nanoparticles [59], and bipyramid gold nanoparticles [60], have been prepared as active SERS substrates (Figure 3). Ma et al. [59] synthesized monodispersed gold nanoflowers using pyromellitic dianhydride-p-phenylene diamine-PPDD under water-based conditions to establish an ultrasensitive SERS method for detecting amantadine in chicken. The limit of detection (LOD) of the method for amantadine was 0.005 ng/mL, the recovery of standard addition was 74.76%–89.34%, and the coefficient of variation was less than 15.04%. Han et al. [51] fabricated silver nanorod arrays as the active SERS substrates via the oblique angle deposition method using a custom-built electron beam evaporation system. The substrate they prepared achieved highly sensitive and reproducible detection of metronidazole and ronidazole. Under alkaline conditions, Sagar et al. [61] successfully synthesized uniformly spherical silver nanoparticles with an average diameter of 40 nm as the active SERS substrate using beta-cyclodextrin as the reducing agent. Using these silver nanoparticles, they developed a rapid on-site detection SERS method for tetracycline residues in milk and water. The LOD of tetracycline in both solutions was as low as 0.01 ppm [61].

Aside from morphology and size, the composition and structure of noble metal nanomaterials also play an important role in the performance of SERS. In general, single-component-based noble metal nanoparticles have poor selectivity and are easily interfered by impurity molecules that results in weak or lost SERS signals, which negatively affects the sensitivity and accuracy of detection results. Two-component-based noble metal nanoparticles with a core-shell structure have been constructed. They can not only retain the physical and chemical properties of the central core and the shell materials but also endow the nanoparticles with some unique properties, such as biocompatibility, monodispersity, and high stability. This construction concept is widely utilized in preparing active SERS substrates [62]. For example, Akshaya et al. [63] proposed a method of stepwise silver reduction on the surface of prefabricated gold nanoparticles to synthesize Au@Ag core-shell nanoparticles. The thickness of the silver shell and the size of the gold core can be adjusted. Sivashanmugan et al. [64] expanded a substrate with a single-metal shell structure into a substrate with a double-metal shell structure. They prepared the active SERS substrate of Au/Ag/Au nanorods via focused ion beam and nanoindentation. These techniques protected the samples from residual contamination and provided a large density of Raman hotspot areas with an enhancement factor of 2.15 × 10^8^ [64].

#### 3.1.2. Hybrid Materials of Noble Metals and Semiconductors as Active SERS Substrates

Although the SERS enhancement effect of noble metals is remarkable, they have certain limitations, such as steep price, poor stability, and low reproducibility, which limit its application in real samples. Semiconductor materials have recently received increased attention as active SERS substrates owing to their unique properties, such as photoelectrocatalytic properties and surface effects [65]. However, the SERS activity of the semiconductor material itself is weak and cannot be used alone as an enhanced substrate. Therefore, semiconductors are combined with noble metal nanomaterials to harness the electromagnetic enhancement mechanism of noble metals and the charge transfer at the interface of semiconductor materials. The synergistic effects of noble metals and semiconductors endow active SERS substrates with notable SERS activity. Huang et al. [66] synthesized Ag/TiO_2_ nanocomposites via a catalytic hairpin assembly strategy. Owing to the surface plasmon resonance of silver nanocubes and the charge transfer effect of TiO_2_, they achieved an excellent Raman spectrum enhancement effect and a highly sensitive detection of targets. Song et al. [67] developed a monodispersed tungsten disulfide quantum dot-modified silver nanosphere (Ag@WS_2_QD) as an active SERS substrate. They synthesized this substrate via a sonication and a hydrothermal route. This substrate exhibited an extremely high Raman enhancement effect on SERS detection, and its enhancement factor was four times higher than that of pure silver nanoparticles.

#### 3.1.3. Hybrid Materials of Noble Metals and MOFs as Active SERS Substrates

MOFs are a class of crystalline porous materials with a high porosity and a large internal surface area [68] In general, a one-pot self-assembly reaction is employed to synthesize the required framework composition and structure by designing the composition of different metal ions and ligands. Owing to their relatively simple preparation, low cost, and excellent properties, such as adjustable structure, controllable functions, multiple active sites, and easy functionalization, MOFs provide a unique platform for SERS detection that has attracted the attention of researchers [69]. Yu et al. [70] reported for the first time that methyl orange molecules adsorbed on the surface of a single component have a SERS effect. However, the SERS enhancement effect of this MOF is unsatisfactory. Therefore, the three-dimensional porous structure and the ultrahigh surface area of MOFs are exploited by combining SERS active noble metal nanoparticles with MOFs that form numerous stable and uniform SERS hotspots with enhanced detection sensitivity. According to the combination of noble metal nanoparticles and MOFs, these hybrid materials can be classified into three categories: (i) noble metal nanoparticles embedded within MOF substrates, (ii) noble metal nanoparticles encapsulated in MOF, and (iii) noble metal nanoparticles modified onto MOFs. Among these structural substrates, the substrate modified with noble metal nanoparticles on MOFs has the best enhancement ability because molecular signals can be directly enhanced at the interface between the noble metal nanoparticles and the MOFs without any hindrance. Jiang et al. [71] developed a highly efficient SERS substrate by in situ synthesis of silver nanoparticles on the surface of a typical MOF, that is, MIL-101 (Fe). They reported that MIL-101 (Fe) provided a large surface area for efficient modification of silver nanoparticles and adsorption of analytes, resulting in a dramatic enhancement of Raman signals.

### 3.2. Quantitative Analysis

The aforementioned active SERS materials to a large extent address the defects of weak Raman signals of analytical targets. In practical applications, the accuracy of quantitative methods is of utmost importance. The most commonly used SERS quantification technique is external standard quantification [72]. In this technique, the Raman signal intensity of the analyte is positively correlated with its concentration. However, owing to the complex matrix of samples, the analyte's concentration has a great impact on the volatility of Raman signals. Furthermore, its contribution to the Raman signal primarily comes from the “hotspot” area of the nanobase material. However, the uniformity of the hotspot of the base material is difficult to control, thus greatly reducing the reproducibility of SERS detection results [73]. Therefore, if SERS is to be used to analyze quantitatively trace substances in actual samples, accurate and reliable quantitative analytical methods must be investigated and developed.

The internal standard method quantitative technology eliminates or minimizes the influence of Raman signal fluctuations and uneven distributions of substrate hotspots and sample matrix by standardizing Raman spectrum signals, thereby improving the accuracy and reliability of detection results [74]. Several researchers have proposed various internal standard quantitative strategies for correcting variations in SERS intensity induced by variations in the physical properties of enhancing substrates [75]. Guo et al. [76] established a quantitative method for analyzing tigecycline in biological samples using silver nanoparticles as the active SER substrate and streptomycin sulfate as an internal standard. The LOD of this method was 2 × 10 − 10 M, and the RSD was 1.6%. However, the internal standard added to the sample usually directly competed with the analyte for adsorption on the enhanced substrate, thus increasing the likelihood of obtaining false-positive results [77].

The embedded internal standard method was developed to reduce the influence of competitive adsorption. The embedded internal standard can exist independently of the substrate structure and does not participate in the target adsorption detection process. However, its Raman signal fluctuations completely reflect the inhomogeneity of the substrate. Zhou et al. [78] designed and synthesized Au@4-ATP@Ag nanomaterials as an enhanced substrate. They used 4-aminothiophenol embedded in the middle of the core-shell structure as an internal standard to correct the Raman signal fluctuations caused by various factors, such as samples and instrument parameters. The LOD of the target molecule was up to 5.0 *μ*M, thereby improving the reliability of quantitative detection results. On the basis of unique spectral shape deformation quantitative theory, Zhang et al. [79] introduced multiple internal standards into SERS quantitative analysis for the first time. They used 2-mercaptobenzimidazole (2 MB) and p-aminothiophenol (PATP) as multiple internal standards. They embedded these standards in Au@Ag core-shell nanoparticles to synthesize Au@2 MB + PATP@Ag as the active SERS substrate. They used Au@2 MB + PATP@Ag to detect quantitatively the phosmet residues on apple skin. Compared with a single internal standard, multiple internal standards provided more characteristic SERS peaks, thereby further improving the efficiency and accuracy of the quantitative results of SERS analysis. The average relative deviation between the quantitative results of the proposed method and those of ICP-MS was about 8%. The embedded internal standard method provides a new idea for accurate quantitative detection of SERS. However, its preparation process is relatively complicated, and the choice of internal standard is limited by the preparation method.

### 3.3. Role of Sample Pretreatment

Although the performance of various types of active SERS substrates is remarkable, owing to the complexity of food matrices, substances with a structure similar to that of the target molecule will compete for adsorption in the hotspot area of the substrate, thereby greatly reducing the detection sensitivity of SERS. Filgueiras et al. [80] found that the carbonyl group of levofloxacin and the hydroxyl group of tetracycline can strongly adsorb on the surface of nanosilver materials, whereas the carbonyl group of benzylpenicillin is weakly adsorbed. When levofloxacin and tetracycline are presented at the same time, directly detecting benzylpenicillin poses a great challenge. In general, the content of antibiotics in food is extremely low (ppb level), and the food sample matrix is complicated. In addition, the SERS technology is only a pure spectrum detection technology without a separation function. Therefore, choosing a suitable pretreatment method to eliminate the interference of complex matrices before detection would substantially improve the selectivity and sensitivity of the SERS technology [81].

The conventional pretreatment technologies for detecting antibiotics in food are liquid-liquid extraction, solid-liquid extraction, and solid-phase extraction [82]. Liquid-liquid extraction is limited by its poor selectivity, cumbersome operation, and consumption of large amounts of organic solvents [83]. Owing to its simple operation, solid-liquid extraction is widely used. Ma et al. [84] preliminarily explored the application of solid-liquid extraction in SERS detection. They established a SERS method for detecting sulfamethazine in aquatic products using ethyl acetate as the extractant and silver nanoparticles as the substrate. They achieved satisfactory results.

Among these preprocessing technologies, solid-phase extraction is currently the most widely used in the detection of antibiotics in food. In this method, the functional groups of the adsorbent material are used to adsorb the target molecule on the surface through interaction forces, such as *π*-*π* interactions, dipole-dipole interactions, ionic bonds, hydrogen bonds, and dispersion force. Afterward, the target molecule is eluted with an eluent or subjected to heating desorption to separate and enrich the target analyte. Crucially, solid-phase extraction can realize automatic batch processing and attain high recovery rate and good reproducibility. However, owing to its low selectivity for the adsorption of target molecules, the traditional solid-phase extraction cannot be effectively applied to extract and enrich trace target compounds in complex samples. With the rapid development of separation technologies in recent decades, some innovative and functional separation technologies have been successfully devised and applied in SERS detection.

Molecular printing technology has been recently applied in sample pretreatment. Gao et al. [85] used chloramphenicol as a template molecule to synthesize molecularly imprinted polymers (MIPs) via “dummy” precipitation polymerization and then combined it with SERS to determine chloramphenicol in milk and honey products. They provided a reliable method for detecting trace levels of chloramphenicol in food systems within 15 min. Moreover, a series of magnetic MIPs (MMIPs) are utilized in the pretreatment of food samples. MMIPs not only have a specific binding function but also possess magnetic properties for further separation. Ekmen et al. [86] successfully prepared surface MIP nanoparticles (MIP@Fe_3_O_4_ NPs) for pretreating malachite green through living/controlled radical polymerization mechanism. They referred to this mechanism as reversible chain transfer catalyzed polymerization. After the target molecules in the sample were specifically identified, captured, separated, and enriched by the MIP@Fe_3_O_4_ NPs, the silicon wafer SERS sensing platform modified with silver dendrites was used to detect the target molecules. Under optimal conditions, the LOD and limit of quantification (LOQ) of the proposed method for detecting malachite green in tap water samples were 1.50 and 4.96 pM, respectively.

Solid-phase extraction based on aptamers have also drawn a great deal of attention in the field of sample pretreatment because they can form various three-dimensional structures through intramolecular interactions, such as “hairpins,” convex loops, pseudoknots, and G-quadruplex structures, which can specifically identify and capture target molecules [87]. Compared with antibodies, aptamers possess unique features: they can be simply synthesized in vitro, and they do not require laboratory animals, they can be easily modified with various tags, and they have good thermal stability with wide temperature and pH ranges [88].

Researchers have also introduced other pretreatment techniques for SERS detection. Chen et al. [89] designed a miniaturized array gas membrane separation device for separating volatile target analytes from matrix impurities. After reabsorption or derivatization, the volatile target analyte was transformed into a substance with a strong SERS response for determination.

In summary, extracting, separating, and purifying the target analytes from complex samples through sample pretreatment to prevent the interference of sample matrixes would further broaden the applications of Raman spectroscopy.

### 3.4. Role of Chemometrics

Scientists have attempted to improve the sensitivity and accuracy of SERS detection in complex matrices by developing various pretreatment technologies and synthesizing different types of enhanced substrate materials. The obtained Raman spectra must be further discovered and analyzed. Chemometrics, which is derived from mathematics and statistics and used to solve practical problems in chemistry [90], is frequently adopted to analyze effectively overlapping Raman spectra to improve the quantitative analysis of SERS accuracy.

In general, when SERS and stoichiometry are combined to conduct quantitative analysis of the target, the SERS signal must be preprocessed by removing fluorescence background interference and reducing the influence of noise to make the characteristic signal more prominent. Furthermore, feature peak from the data is extracted from the preprocessed spectrum. Finally, a predictive model is established to analyze the target qualitatively or quantitatively [91].

In chemometric analysis, the choice of mathematical models for calibration set samples are critical to the accuracy of results. The selected mathematical model should have the ability to correlate the content of a known analyte in the calibration set with the characteristics of the SERS spectral data, and the model can also be used to predict the content of the analyte in an unknown sample. Moreover, the range of the content of the analyte in the calibration set sample should be greater than that of the analyte in the predicted sample so that the model has a strong universal applicability. Many types of models are used in SERS quantitative analysis, such as multiple linear regression (MLR) [92], principal component regression [93], partial least squares [94], artificial neural networks [95], and least squares-support vector machine [96]. Lee et al. [97] intercepted SERS spectral signals of 400-1,800 cm^−1^ in the quantitative detection of monensin, decoquinate, and lasalocid. They adopted multiple linear regression (MLR), partial least squares regression (PLSR), and principal component regression (PCR) to establish a quantitative prediction model of antibiotics in samples. These models achieved a high accuracy in predicting the concentration of antibiotic standard solutions. The prediction accuracy of MLR within the low concentration range was comparable to that of HPLC. In predicting spiked samples, the accuracy of MLR and PLSR was still high, whereas PCR performed poorly with unsatisfactory accuracy. However, the models could not adequately predict spiked samples with a low concentration, and their prediction error was large largely because of the strong noise interference caused by fluorescence signal background and SERS substrate physical factors in complex systems that reduced the prediction accuracy of the models.

To reduce the influence of noise and improve the accuracy of prediction models, researchers have focused on optimizing the algorithms. Liu et al. [98] used adaptive iteratively reweighted penalized least squares to preprocess raw SERS data. Specifically, they adjusted adaptively and iteratively the weight of the residual sum of squares between the fitting baseline and the original signal. Subsequently, they employed the moving window partial least squares algorithm to establish a prediction model of voriconazole content in samples. The correlation coefficient of the model when the concentration of voriconazole was 0.003–200 *μ*g/mL was 0.99, its RMSEP was 2.98, and its prediction accuracy was satisfactory. Hong et al. [99] constructed a predictive model for simultaneous detection of enrofloxacin and ciprofloxacin in drinking water using the alternate least square algorithm. They performed principal component analysis to reduce the dimensionality of Raman spectroscopy data and then extracted characteristic factors to establish the model. The LOQ of the model achieved ppm level, and the RSD was less than 10%.

The development of SERS quantitative analytical methods is largely attributed to improvements in chemometric analysis and multivariate analysis that may provide new solutions for the detection and monitoring of antibiotics.

### 3.5. Functional Integration

Although SERS is considered a potential single-molecule detection method, it does not have the function to separate target molecules from complex sample matrices, a crucial defect that limits its application in trace analysis [100]. Thus, to overcome the nonspecificity of SERS in antibiotic detection, researchers have evaluated specific target capture media to explore the potential of SERS in terms of selectivity. Several methods that can specifically identify targets are integrated with SERS to enhance the selectivity of SERS for trace analytes.

Immunochromatography is a method that combines chromatographic methods with antigen-antibody immunoreactions for specific detection of target molecules. However, this method cannot be used for quantitative analysis. Integrating SERS with immunochromatography (SERS-ICA) not only solves the quantification problem of immunochromatography but also improves the selectivity and sensitivity of SERS. Sun et al. [101] were the first to use SERS-ICA for the specific quantitative analysis of trace phenylethanolamine A. They have also applied SERS-ICA in detecting other targets. For instance, they used 4-mercaptobenzoic acid (MBA) as the Raman reporter and synthesized Ag^MBA^@SiO_2_-Ab as the probe to establish a fast and convenient SERS-ICA method for on-site detection of diclofenac residues in environmental water samples (Figure 4). The LOD of diclofenac was 0.07 pg mL^−1^, and the RSD was less than 6.0%. Moreover, no cross-reaction occurred with other compounds. The high sensitivity and high accuracy of this method indicated that the “sandwich” structure of SERS-ICA has broad application prospects [102]. On the basis of similar principles and procedures, they used colloidal gold as a Raman-enhanced substrate. They labeled it with MBA and monoclonal antibody to synthesize a double-functionalized Ab-Au-MBA as an immunoprobe. With Ab-Au-MBA immunoprobe, SERS-ICA was successfully applied for the detection of 3-amino-5-methylmorpholino-2-oxazolidinone in tissues and urine [103]. Interestingly, this method does not require derivatization, and the detection can be completed within 15 min, displaying high specificity, reproducibility, and stability. Shi et al. [54] employed 4-aminothiophenol (PATP) as the Raman probe to synthesize AuNPs-PATP immunoprobes and constructed a rapid detection method based on SERS-ICA for detecting neomycin in milk. The LOD of this method was 0.216 pg/mL, and no cross-reactivity occurred between the assay and other compounds, demonstrating that the assay had high specificity. Li et al. [104] extended the single-component detection to multiple-component simultaneous detection. The LOD was 10^−5^ ppb, and the sensitivity was three to four times higher than that of ELISA and ICA. However, SERS-ICA also has shortcomings. Some antibodies are difficult to prepare, the antibodies have unstable properties, and the method has poor reproducibility, all of which limits its application.

Aptamers, which are also known as “chemical antibodies,” are DNA or RNA fragments screened via systematic evolution of ligands by exponential enrichment technology. They can specifically bind to target molecules through hydrogen bonding, electrostatic interactions, and conformational complementation to achieve enrichment and separation with high specificity, high affinity, and easy chemical synthesis and modification [105]. Compared with ICA, aptamers have a wider range of applications because they are more stable and have a better reproducibility. Therefore, aptamers combined with spectroscopy are widely used in detecting complex samples, including food [106], medicine [107], and environmental sample [108]. Jiang et al. [109] proposed a SERS method with an aptamer sensor for detecting kanamycin in milk. As shown in Figure 5, the DNA probe is embedded on the surface of gold nanoparticles via sulfhydryl end modification and then encapsulated with a silver shell. The aptamer DNA with the Raman signaling molecule Cy3 is hybridized with the probe DNA through complementary base pairing to synthesize the kanamycin aptamer sensor Au@Ag NPs-dsDNA. When kanamycin is present in the sample, the aptamer DNA of kanamycin detaches from the surface of Au@Ag NPs, resulting in the weakening of the Raman signal of Cy3 on the surface of Au@Ag NPs. On the basis of this principle, Jiang et al. [109] established the quantitative detection method. Their method had high sensitivity with an LOD of 0.90 pg/mL and had good linearity from 10 *μ*g/mL to 100 ng/mL. Zhuang et al. [110] used Cy5-labeled DNA as a Raman signal generator and a specific recognition probe embedded in Au@Ag NSs to establish a highly sensitive and specific detection method for chloramphenicol. The LOD was 0.19 pg/mL, and this method did not require a complicated self-assembly process to achieve ultrasensitive detection of this antibiotic.

The aforementioned antibodies and aptamer probes have outstanding performance in terms of specificity. However, in detecting analytes with a low molecular weight, these two methods are largely inaccurate because the recognition sites of small molecules hinder the development of the Sandwich structure between small-molecule probes and capture molecules [111]. In recent years, MIPs synthesized via molecular imprinting technology that have specific recognition functions for template molecules have attracted increased attention.

In general, MIPs are also called “lock-key” technology. As shown in Figure 6, the template molecule, the functional monomer, the cross-linking monomer, and the initiator are polymerized to form a complex. After cleaning the template molecules from the complex, a cavity complementary to the template molecules is formed for specific recognition and capture of the template molecules [112]. Compared with antibodies and aptamers, MIPs possess a higher physical strength, better stability, longer service life, and inertness to many chemicals. The combination of MIPs and SERS has a wide application prospect in the detection of complex matrices. Carrasco et al. [113] prepared multibranched gold-silica-MIPs (bAu@mSiO_2_@MIP) as SERS probes for ultrasensitive detection of enrofloxacin. After enrofloxacin was combined with the recognition site in the MIPs, the plasmon resonance caused by the nearby multibranched gold nucleus greatly enhanced the Raman signal of the target. Its LOD reached 1.5 nM, and no other potential species that can cause interference was found. Similar methods have been successfully used in the detection of patulin [114], cloxacillin [115], and other antibiotics. However, during the preparation of MIPs, removing all template molecules from the polymer network is difficult. Mosbach et al. [116] noted that at least 5% of the template molecules remains in the polymer network structure after elution, which would generate obvious background interference signals in the detection, thereby severely limiting the detection of trace and ultratrace substances by MIPs-SERS.

On the basis of MIPs, the dummy molecular imprinting technique has been proposed. Its core strategy is to use molecules similar to the detection target molecule as template molecules, which addresses the aforementioned defects of MIPs. Chen et al. [117] utilized abietic acid as a dummy template molecule and prepared Ag@dummy MIPs as a SERS substrate for the identification and detection of crystal violet. No interference signal was generated when the concentration of crystal violet was 10^−9^ mol/L. In another study, they used a similar method to synthesize Ag@dummy MIPs-SERS substrate using carbendazim as a template to establish a SERS detection method for benzimidazole. Its LOD was 10^−8^ mol/L, and its sensitivity was satisfactory. They also evaluated the reusability of Ag@dummy MIPs. The fingerprint peaks of the analyte slightly decreased after using it four times, but the intensity of the characteristic peaks remained obvious. Therefore, Ag@dummy MIPs can be reused [118]. This feature not only reduces the cost of testing but also saves time on preparing materials, which are crucial in practical applications.

## 4. Future Trends

SERS has a strong application potential and high practical value in the field of food safety evaluation because of its technical advantages, such as fast detection, resistance to water interference, and its ability to provide fingerprint structure information of the target [119]. However, this method also has many limitations and deficiencies when applied in detecting complex sample matrices. Thus, SERS must be further optimized and improved.

First, the Raman signal intensity of trace analytes in samples is very weak, and it cannot be directly measured. Therefore, because of the complexity and diversity of food samples, Raman signal enhancement substrate materials with a uniform morphology and stable physical properties must be synthesized. Although some substrate materials with a good reproducibility and a high sensitivity have been commercialized to meet testing needs, their high price has severely restricted their widespread use in food safety evaluation. With the development of nanotechnology, reducing the cost of substrate materials will become the focus of future research. In addition, SERS is a spectroscopic technology that does not have a separation function. Therefore, functionalized substrates that can specifically identify and capture target objects are important to the application of SERS in the detection of trace analytes in food.

Second, a fluorescence effect is generated when laser irradiates food samples, the intensity of which is often several orders of magnitude stronger than that of the Raman signal, thereby causing strong background interference and even completely annihilating the characteristic Raman signal of the target. Therefore, reducing the fluorescence background interference is the key to the sensitive and accurate detection of antibiotics in food by SERS. Researchers primarily deal with these problems from two aspects, that is, improving both the hardware and software of equipment. In terms of hardware, various methods, such as confocal microscopy and pulse technology, are used, but the impact of the detection environment noise still cannot be eliminated. In addition, as the complexity of the instrument system increases, electronic and optical systems may cause greater noise. Therefore, the hardware optimization effect is limited. In terms of software, the introduction of chemometrics can make the characteristic signal of the test object more prominent, as well as enable the removal of background interference and reduction of the influence of noise, thereby remarkably improving the sensitivity of detection. With the advent of the “Data Era,” processing Raman spectroscopy data will move toward automation, artificial intelligence, and cloud computing. This development would allow the effective application of SERS in food inspection. Finally, the development of low-cost and portable SERS equipment for field testing is also the main research direction.

## 5. Conclusions

This article reviewed the progress that has been achieved in the research on SERS in the detection of antibiotic residues in food. This article discussed the basic principles of SERS, active SERS substrates, sample pretreatment, quantitative methods, application of chemometrics in SERS, and functional integration. This article also laid out prospects for the future development of SERS. The combination of SERS and other technologies can remarkably improve the detection performance of SERS with strong application potential in complex food matrices. However, as a fast and sensitive detection technology, SERS requires further development to realize its effective application in detecting antibiotics in food.

## Figures and Tables

**Figure 1:** Schematic of the general pathway chain illustrating the use of antibiotics in farm animals/crops and the subsequent employment of SERS testing of various antibiotic-contaminated foods.

**Figure 2:** Illustration of SERS mechanism [25].

**Figure 3:** Scanning electron micrographs of (a) gold nanostars [57], (b) silver nanodendrites [58], (c) bipyramid gold nanoparticles [59], and (d) flower-like gold nanoparticles [60].

**Figure 4:** (a) Schematic of the preparation of the immunoprobe (AgMBA@SiO_2_-Ab NPs). (b) Assembly of the ICA strip, and schematic of SERS-based ICA for DCF [102].

**Figure 5:** Schematic of the SERS-based method for KANA detection using double-strand DNA aptamer-bonding Au@Ag NPs [109].

**Figure 6:** Overview of MIP imprinting [112].

**Table 1:** Different analytical techniques for the determination of antibiotics in food.

Analytical method	Tentative detection levels	Remarks	Ref.
Surface-enhanced Raman spectroscopy (SERS)	0.11 *μ*M	(i) Detection of 2-mercapto-5-methyl-1,3,4-thiadiazole in real milk	[8]
		(ii) Nonselective	
		(iii) Low sample consumption and fast response	
		(iv) Simple operation, high sensitivity, strong selectivity, less interference from water	
		(v) Can be used for molecular structure analysis	
		(vi) On-site determination	
Capillary electrophoresis	4.1–6.3 ng/mL	(i) Detection of ciprofloxacin in chicken muscle	[9]
		(ii) Fast analysis and high precision	
		(iii) Used with a mass spectrometer, a diode array detector, and a fluorescence detector	
		(iv) Sensitivity and repeatability must be improved	
Electrochemical techniques	0.003 *μ*M	(i) Detection of sulfanilamide in milk	[10]
		(ii) Simple operation, high sensitivity, low cost	
		(iii) Low stability	
		(iv) In samples with complicated matrices, problems with repeatability may occur due to deterioration of electrodes	
Liquid chromatography-mass spectrometry	1.46–15.5 ng/kg	(i) Detection of sulfonamides in aquaculture	[11]
		(ii) The most authoritative method in antibiotic detection	
		(iii) High sensitivity and selectivity	
		(iv) Requires expensive equipment	
		(v) Sample preparation is time consuming	
		(vi) Difficult to detect on site	
Immunochromatography	0.6 ng/mL	(i) Detection of furazolidone in pork, shrimp, and eggs	[12]
		(ii) High sensitivity and specificity	
		(iii) Simple operation, fast detection, and low price	
		(iv) Suitable for on-site detection	
		(v) Qualitative or semiquantitative detection	
		(vi) False-positives may be obtained because of the interference of complicated matrices	
Enzyme-linked immunosorbent assay (ELISA)	2.42–4.88 *μ*g/kg	(i) Detection of quinolones, tetracycline, lincomycin, and streptomycin in milk	[13]
		(ii) Simple operation, fast, high sensitivity, and high specificity	
		(iii) Prone to false-positives by the interference of autoantibodies and heterophile antibodies	
		(iv) Poor repeatability	
		(v) Greatly affected by detection time and temperature	
		(vi) High sensitivity and specificity	
		(vii) Simple operation, fast detection and low price	
		(viii) Suitable for on-site detection	
		(ix) Qualitative or semiquantitative detection	
		(x) False-positives may be obtained because of the interference of complicated matrices	

**Table 2:** A summary of various antibiotic drugs that have been analyzed in foods by using SERS with various active substrates.

Antibiotics	Analytes	Substrates	Matrixes	Limit of detection	Ref.
Sulfonamides	Sulfamethoxazole	RGO/Ag-coated alloy fibers	Tissue mimic	4.4 ng·cm^−3^	[32]
	Sulfadiazine				
	Sulfamerazine	AuNPs	Muscle foods	100 ppb	[33]
	Sulfamethazine				
	Sulfamethoxazole	Ag NPs	Human urine	1.7 *μ*g/mL	[34]
Quinolones	Levofloxacin	Au@Ag core-shell nanorods	Food animal products	0.37 ng/L	[35]
	Enrofloxacin	Dendritic Ag NPs	50% ethanol solution	20 ppb	[36]
	Ciprofloxacin		Hydrochloric acid solution		
	Moxifloxacin	Commercial substrates	Animal urine	0.085 *μ*g/mL	[37]
	Benzylpenicillin	Ag NPs	Water	1 × 10^−7^ mol/L	[38]
	Carbenicillin	Ag NP	Drinking water samples	0.63 × 10^−8^ mol/L	[39]
	Danofloxacin	Ag-TiO2	Water	3.16 × 10^−11^ mol/L	[40]
	Enoxacin			3.15 × 10^−10^ mol/L	
	Penicillin G sodium	AgNPs/AC	Aqueous solution	5.09 × 10^−11^ M	[41]
	Ampicillin	Ag NPs	Milk	10 ppb	[42]
	Amoxicillin	Three-dimensional ZnO/Ag-9	Water	10^−9^ M	[43]
Chloramphenicols	Chloramphenicol	Au@Ag nanoparticles	Aquatic products	0.36 ng/mL	[44]
	Thiamphenicol			0.20 ng/mL	
	Florfenicol			0.78 ng/mL	
Tetracyclines	Tetracycline	MNs-aptamer/cDNA-APS	Deionized water	0.001 ng/ml	[45]
	Doxycycline	OTR202 and OTR103	Duck meat	1.346 mg/L	[46]
Cephalosporins	Ceftriaxone	CaCO3-CuNP	Deionized water	5 *μ*M	[47]
	Cefazolin	CuNPs	Human urine	7.5 *μ*g/mL	[48]
	Cefoperazone				
	Ceftriaxone				
Lincomycins	Kanamycin	Graphene-gold nanocomposite	Drinking water, orange juice, and milk	0.75 nM	[49]
		Au@Ag NPs-4MBA	Milk	142 pg/mL	[50]
Methylimidazoles	Metronidazole	Ag NRs	Ultrapure water	10 *μ*g/mL	[51]
	Ronidazole			1 *μ*g/mL	
	Metronidazole		Tap water	10 *μ*g/mL	
	Ronidazole			10 *μ*g/mL	
	Metronidazole		Metronidazole lake water	50 *μ*g/mL	
	Ronidazole			10 *μ*g/mL	
	Metronidazole		Swamp water	50 *μ*g/mL	
	Ronidazole			10 *μ*g/mL	
	Metronidazole		Environmental soil	10 *μ*g/mL	
	Ronidazole			2 *μ*g/mL	
Macrolides	Erythromycin	Ag NPs	Mixture of distilled water and ethanol	2.38 × 10^−6^ mol/l	[52]
Oxytetracycline	Oxytetracycline	AgNPs	Honey and other food samples	5 ppb	[53]
Aminoglycosides	Neomycin	AuNPs	Milk	0.216 pg/mL	[54]
Nitrofurans	Furadantin	Au-NPs	Food	5 ppm	[55]
	Furaltadone				

## Data Availability

All data generated or analyzed during this study are included within the article.
